The article "Influence of Nurse-Led Health Education on Self-Management Ability, Satisfaction, and Compliance of Elderly Patients with Chronic Obstructive Pulmonary Disease Based on Knowledge, Belief, and Practice Model" was retracted in 2023. Reasons: signs of a paper mill; compromised peer review; unreliable results or conclusions.

# Influence of Nurse-Led Health Education on Self-Management Ability, Satisfaction, and Compliance of Elderly Patients with Chronic Obstructive Pulmonary Disease Based on Knowledge, Belief, and Practice Model

**DOI:** 10.1155/2022/1782955

**Published:** 2022-08-08

**Authors:** Wenyan Hu, Tingyan Li, Shenglong Cao, Yongping Gu, Liyan Chen

**Affiliations:** ^1^Linping Campus, The Second Affiliated Hospital of Zhejiang University School of Medicine Pulmonary and Critical Care Medicine, Hangzhou, China 311100; ^2^The Second Affiliated Hospital Zhejiang University School of Medicine, Hangzhou, China 311100

## Abstract

**Objective:**

Knowledge, belief, and behavior model (knowledge-attitude-practice (KAP)) is known as a cognitive model. Health education is important to the prognosis of patients, including chronic obstructive pulmonary disease (COPD) patients. However, the investigation regarding health education based on the KAP model is few. Thus, this work is aimed at analyzing the influence of nurse-led health education on self-management ability, satisfaction, and compliance of elderly patients with COPD based on knowledge, belief, and practice model.

**Methods:**

60 elderly patients with COPD cured in our hospital from January 2019 to April 2021 were enrolled for the study. The patients were randomly assigned to control group (*n* = 30) and study group (*n* = 30). The former group received routine nursing, and the latter group accepted health education based on “knowledge, belief, and practice” model. Finally, the scores of nursing satisfaction, KAP score, compliance rate, self-management level, pulmonary function, and life quality were compared in the two groups.

**Results:**

The nursing satisfaction of the study group (100.00%) was higher than that (83.33%) of the control group (*P* < 0.05). The scores of knowledge, attitude, and behavior were remarkably higher in the study group than in the control group after nursing (*P* < 0.05). Moreover, KAP scores also significantly increased in the study group after nursing. The compliance rate of the study group (93.33%) was higher than that of the control group (66.67%) (*P* < 0.05). After nursing, the scores of symptom management, daily life management, emotion management, information management, and management efficiency were higher in the study group than in the control group (*P* < 0.05). In addition, pulmonary functions were improved in the two groups following nursing. Compared with the control groups, the 6 min walking distance, FEV1%, and FEV1/FVC% were higher in the study group (*P* < 0.05). After nursing, the scores of life quality were reduced in the two groups. The scores of physiological function, psychological function, social function, and health self-cognition were lower in the study group than in the control group (*P* < 0.05).

**Conclusion:**

Based on the model of knowledge, belief, and practice, nurse-led health education can successfully enhance the self-management ability, satisfaction, and compliance of elderly COPD patients.

## 1. Introduction

Chronic obstructive pulmonary disease (COPD) causes progressive airflow obstruction, usually due to airway and/or alveolar abnormalities caused by exposure to toxic gases or particles [1]. COPD has high rates of morbidity, mortality, and disability and imposes a burden on individuals, families, and society. The prevalence of COPD is increasing year by year and tends to be younger [2], but the elderly are still the main disease group. In the context of aging in China, the number of COPD patients is increasing year by year. So far, there is no complete cure for COPD in the world, and the main clinical treatment strategy is to delay the development of the disease through drug treatment and nondrug treatment. The commonly used drugs are glucocorticoid, bronchodilator, antiasthmatic, and expectorant. However, medication is not the end point of COPD therapy. Long-term medication commonly confers drug resistance, thus affecting disease control [3].

Elderly patients with COPD lack health knowledge and have anxiety and bad living habits, such as unreasonable diet, smoking, and alcohol addiction, and can lead to various complications. A previous study found that the life quality of elderly COPD patients was lower in all aspects in comparison with healthy controls [4]. Therefore, the nurses need to continuously increase health education for patients with liver cirrhosis, which is very important to avoid or reduce complications. Health education has clear goals and objectives. It is necessary to achieve goals and objectives through feasible measures to evaluate, analyze, and feedback on the effect of education. With the continuous development of nursing research, the methods, contents, and forms of clinical nursing health education are also constantly improving [5].

The knowledge, belief, and action model of health education is a behavior change theory proposed by Dr. Gcust in the 1960s [6]. Knowledge, belief, and behavior model (knowledge-attitude-practice (KAP)), known as a cognitive model, is a more mature model of behavior change. Among them, knowledge, namely, knowledge and learning, is the foundation. Belief and attitude are motivation. Practice is the process of generating healthy behavior and eliminating harmful behavior [7]. The model of knowledge, belief, and practice was first reported in the 1980s in China. At present, it has been gradually carried out nursing management and health education in China; however, the research on health education based on KAP model is still relatively few [8]. The aim of this study was to build a “knowledge, belief, and practice” health education model for elderly patients with COPD.

## 2. Patients and Methods

### 2.1. General Information

During January 2019 to April 2021, 60 elderly patients with COPD cured were enrolled for the study in our hospital. The patients were discretionarily assigned into control group (*n* = 30) and study group (*n* = 30). The former group accepted routine nursing care, and the latter group accepted health education of “knowledge, belief, and practice mode.” The age of patients in the control group ranged from 61 to 90 years old with an average of 81.29 ± 4.23 years old, including 18 males and 12 females. The course of disease is 2-10 years with an average of 7.03 ± 2.05 years. In the study group, the age ranged from 60 to 91 years old with an average of 81.34 ± 3.29 years, including 16 males and 14 females. The course of disease ranged from 2 to 11 years with an average of 7.12 ± 2.09 years. There exhibited no statistical significance in the general data. Informed consent was obtained from all the patients in this study, which was permitted by the Medical Ethics Association at our hospital. This study was a single blind test.

Selection criteria are as follows: (i) age ≥ 60 years old, (ii) meeting the diagnostic criteria of chronic obstructive pulmonary disease (revised in 2021) [9], (iii) grades II-III of lung function, (iv) stable condition and clear consciousness, and (v) patients with informed consent to the trial.

Exclusion criteria are as follows: (i) patients with severe chronic diseases, (ii) patients with a history of stroke or dementia, (iii) patients with motor dysfunction, (iv) patients with long-term use of drugs that may cause anxiety and depression, and (v) all the patients who were included in the experiment.

### 2.2. Treatment Methods

The patients in the control group accepted routine nursing in the department, and the patients in the study group received a nurse-led health education based on knowledge, belief, and practice model. The specific measures were as follows:

1. Analyzing the physical, mental, family, and social conditions of the patients in the experimental group by questionnaire. Their knowledge, belief, and behavior (KAP) about COPD-related knowledge were investigated, and health records were established for one-to-one individualized intervention guidance
2. The intensive teaching was performed to educate patients about the etiology, risk factors, definition, epidemiology, common symptoms, prognosis, and treatment principles of COPD
3. Respiratory rehabilitation exercise. The exercises including walk training were performed based on the previous methods [10]
4. Distributing education manuals: compiling and distributing health education manuals with pictures and texts to facilitate patients' understanding and implementation
5. According to the health records of each patient, telephone visit was carried out every two weeks for 10-30 minutes. At the same time, the effect of intervention was evaluated, and the causes for noncompliance were analyzed. Finally, the education program was evaluated

### 2.3. Observation Index

#### 2.3.1. Satisfaction

Based on the literature review [11] and expert discussion, we designed 10 questionnaires to measure patients' follow-up satisfaction. Then, the satisfaction of follow-up management mode, health education, medical nursing service, appointment registration process, and so forth were assessed. It is assigned into four levels: very pleased, pleased, general, and displeased. Satisfaction rate = (number of very satisfactory cases + satisfactory cases + general cases)/total number of cases × 100%.

#### 2.3.2. Knowledge Belief and Practice Level

Knowledge, belief, and practice levels were analyzed referring to the relevant literature [12] and then discussed by professionals. We adopted the self-designed COPD knowledge, belief, and practice questionnaire, and its contents included disease-related knowledge, attitude, and behavior. It was used to assess the changes in knowledge, belief, and practice before and after health education. There were three types of options, including correct, incorrect, and uncertain, in the knowledge section of the questionnaire (16 items). Finally, one point was given for correct answers and zero for incorrect or unclear answers. The alternative answers of attitude (2 items) were assigned into three grades, representing negative determination, uncertainty, and negative scores, with 2, 1, and 0 points, respectively. The behavior part (6 items) took yes or no, no as alternative answer with 1 score for the correct answer and 0 for the wrong answer.

#### 2.3.3. Compliance

At discharge, the treatment compliance of patients was evaluated by analyzing the compliance in medication compliance, regular exercise, and healthy diet by nursing staff. The evaluation results were assigned into three categories, including complete compliance, compliance, and noncompliance. Complete compliance indicated that patients could fully implement doctor's advice and actively cooperated with treatment; compliance indicated that patients could basically follow medical instructions and occasionally needed supervision and reminders; noncompliance was basically unable to carry out doctor's orders, or even resisted treatment. The evaluation of treatment compliance was performed referring to the previous study [13]. Compliance rate = (number of patients with complete compliance + number of patients with compliance)/total number of cases × 100%.

#### 2.3.4. Self-Management Scale

The patient's self-management ability was evaluated before (admission) and after nursing (discharge) according to the COPD self-management scale [14]. Self-management scale included symptom management, daily life management, emotion management, information management, and self-management efficacy management. The score of each item was 1-5 points with a total score of 51-255. The overall Cronbach's alpha coefficient of the scale was 0.92. Cronbach's alpha coefficient of each factor was 0.82-0.87, and the CVI value is 0.9015.

#### 2.3.5. Pulmonary Function Index

The pulmonary function indexes were measured before (admission) and after nursing (discharge). The pulmonary function of the two groups was measured using Germany MasterScreen PFT pulmonary function instrument. Finally, the ratio of forced expiratory volume to forced vital capacity (FEV1/FVC) at the first second and the percentage of FEV1 in the predicted value were determined.

Six-minute walk test (6minuteswalktest6MWT): the test site was registered in the open area of the hospital corridor or outdoor. The return distance was 30 meters, and the inflection point should be marked every 3 meters. Explain the requirement and significance of this examination to the patient before the trial begins. To get the patient's cooperation, the patients were asked to walk as fast as possible within 6 minutes. If you felt uncomfortable, you can have a rest and wait until you feel better before walking. Medical staff gave verbal encouragement every minute. Borg scores were performed before the trial to determine the level of dyspnea at rest.

#### 2.3.6. Life Quality Scale

Referring to the previous literature [15], the quality of life survey scale was designed to assess the improvement of patients' life quality in this study. Life quality was evaluated before nursing (admission) and after nursing (discharge), including four subscales: physical, psychological, social, and health self-awareness with a total of 29 items. The scale was rated from 1 to 5. Cronbach *α* coefficient was between 0.79 and 0.91.

### 2.4. Statistical Analysis

Using the SPSS21.0 statistical software, we examined measurement data by normal distribution and variance homogeneity analysis to meet the requirements of normal distribution or approximate normal distribution, which is shown by ($\bar{x}\pm s$). *P* < 0.05 was considered statistically remarkable when comparing the two groups using a *t*-test or *χ*^2^ test.

## 3. Results

### 3.1. Comparison of Nursing Satisfaction

As shown in Figure 1, 22 patients were very pleased, 7 patients were pleased, 1 patient was general, and 0 patient was displeased in the research group, and the satisfaction rate was 100.00% (*P* < 0.05). In the control group, 13 patients were very pleased, 8 patients were pleased, 4 patients were general, and 5 patients were displeased, and the satisfaction rate was 83.33%. Thus, the nursing satisfaction of the study group was higher than that of the control group (*P* < 0.05).

### 3.2. KAP Score Comparison

The KAP scores of patients increased after nursing, and the difference in KAP scores before and after nursing in the study group exhibited statistically significant (*P* < 0.05). The scores of knowledge, attitude, and behavior were higher in the study group than in the control group following the nursing (*P* < 0.05). All the data are indicated in Table 1.

### 3.3. Compliance Comparison

The compliance rate of patients was remarkably higher in the study group than in the control group. In the study group, 15 cases were completely compliant, 12 cases were compliant, and 3 cases were discompliant, and the total compliance rate was 93.33% (*P* < 0.05). In the control group, 8 cases were completely compliant, 12 cases were compliant, and 10 cases were discompliant, and the total compliance rate was 66.67% (*P* < 0.05). All data results are indicated in Figure 2.

### 3.4. Comparison of Self-Management Level

After nursing, the self-management scores of patients were remarkably enhanced in the two groups. After nursing, the scores of symptom management, daily life management, emotion management, information management, and management effectiveness were remarkably higher in the study group than in the control group (*P* < 0.05). All the results are indicated in Table 2.

### 3.5. Comparison of Pulmonary Function

After nursing, the pulmonary functions were enhanced in the two groups. Compared with the control groups, the 6 min walking distance, FEV1%, and FEV1/FVC% were higher in the study group (*P* < 0.05). All data results are indicated in Table 3.

### 3.6. Comparison of Quality of Life Scores

After nursing, the scores of life quality were decreased in the two groups. The scores of physiological function, psychological function, social function, and health self-cognition were lower in the study group than in the control group (*P* < 0.05). All the data results are indicated in Table 4.

## 4. Discussion

Chronic obstructive pulmonary disease (COPD) causes progressive airflow obstruction, usually due to airway and/or alveolar abnormalities caused by exposure to toxic gases or particles [16]. COPD has high rates of morbidity, mortality, and disability, which poses a burden on individuals, families, and society. In order to alleviate clinical symptoms and improve lung function of patients, lung rehabilitation exercise has become a core part of the management of stable COPD patients, but the compliance of COPD patients is often not ideal due to various reasons [17]. Therefore, it is necessary to analyze the status and influencing factors of lung rehabilitation exercise compliance in COPD patients, so that medical staff can adopt effective management strategies.

Health education is part of the work of medical staff to impart health knowledge and disease management techniques to society, families, and individuals through appropriate educational means [18]. Health education can improve patients' compliance with treatment, change bad lifestyle, and reduce the rate of rehospitalization [19, 20]. Traditional health education is often performed by health care staff through oral education or distribution of health education prescriptions for basic and simple health knowledge education [21]. When the level of educational knowledge and belief of elderly COPD patients is insufficient, it will affect the compliance of patients with health behavior changes and disease prevention and delay the implementation of postoperative lung rehabilitation, thus affecting the prognosis of patients [22, 23]. With the development of medicine and science and technology, medical staff have taken a variety of health education for elderly COPD patients recently in order to improve patients' health knowledge and compliance behavior. The application of health education pathway can improve patients' knowledge of lung rehabilitation, strengthen the control of disease risk factors, and prevent and control the incidence of complications [24, 25]. Srinivasan et al. took targeted education and nursing care for elderly COPD through phased health education, which could effectively reduce patients' negative emotions and promote their sleep quality [26]. Some scholars have carried out phased health education for patients and their families during hospitalization and after discharge and achieved good results [27]. The health education can be carried out on elderly COPD [28]. The reflective education makes patients realize that unhealthy lifestyle is an important cause of disease to improve patients' healthy life and medication compliance, which is consistent with the results of Ahuja et al. [29]. At present, the incidence of elderly COPD in China is on the rise, coupled with the uneven distribution of medical resources. It can effectively reduce the out-of-hospital time delay of elderly COPD patients after health education for community residents [30]. In addition, domestic scholars used multicultural nursing education, integrated health education, multidisciplinary education model, authorization theory education, and feedback health education to educate elderly patients with COPD. The results showed that good results were achieved in life quality, negative emotion control, and hospital satisfaction [31–33]. The propaganda and education methods of WeChat group, official account, and mobile medical platform also attach importance to the rehabilitation education of patients with coronary heart disease. They can send text, audio, video, and other materials to make up for the shortcomings of traditional health education. Some mobile medical services can also monitor patients' heart rate, exercise energy consumption, and other functions. The content guidance of cardiac rehabilitation based on evidence-based and expert consensus makes the content of rehabilitation health education for patients with coronary heart disease more comprehensive, scientific, and standardized [34].

Educating people about health care is a process and activity that helps them learn about health concepts, gain knowledge about health care, and enhance their personal health. The theory of knowledge, belief, and behavior (abbreviation of knowledge, belief, and behavior) is also known as KAP theory (KABP or KAP) [35, 36]. It is the continuation of the application of cognitive theory to health education. The knowledge, belief, and behavior (KBB) theory proposes that health knowledge and information are integral to forming positive and correct beliefs and attitudes and to changing health-related behaviors. Beliefs and attitudes are the driving force of behavior change [37, 38]. Patients have to go through a series of processes from acquiring knowledge to behavior. In this process, many factors can affect the smooth transformation and maintenance of knowledge to behavior. Any one of these factors can lead to behavior change. Only when patients think positively about knowledge and gradually form beliefs, it is possible to take a positive attitude to form healthy behaviors [39, 40]. In the traditional way of health education, we only pay attention to the transmission of health information. Developing healthy behaviors and getting rid of harmful behaviors can only be achieved when people have understanding of health knowledge and establish positive attitudes and beliefs. It can be expressed as three continuous processes, namely, knowledge “belief” behavior [41]. Knowledge (knowledge and learning) is the foundation, belief (belief and attitude) is the motivation, and action (promoting healthy behavior) is the goal. COPD patients have a long course of disease and repeated attacks of disease, which brings a heavy economic burden to the family and society [42]. Nurse-led health education based on knowledge, belief, and practice is a scientific nursing method. Its core idea is “people-oriented” and “patient-centered,” which is more humanized than traditional education. It is more helpful to improve the physical and mental state and life quality of patients. Cognition in the theory of knowledge, belief, and practice is the basis of follow-up action. The formation of health beliefs is the key for patients to accept and adopt health advice and develop healthy living habits. In the knowledge, belief, and practice health education model, patients can master more health knowledge; learning efficiency and learning initiative will be greatly improved, which will be of great benefit to the improvement of their condition and life quality. At present, there exhibits no specific targeted therapy for COPD, and traditional drug therapy alone can no longer meet the needs of patients. More and more professionals at home and abroad agree on health education for patients and their families. It is proposed that nondrug therapy is a main supplementary treatment method for COPD patients in the advanced stage, which can successfully treat patients and prevent further deterioration, including rehabilitation, smoking cessation, long-term oxygen therapy, and noninvasive mechanical ventilation [43]. Fujino et al. followed up 56 COPD patients with respiratory muscle rehabilitation training for 1 year [44]. The number of hospitalizations and colds was remarkably reduced, and the indicators of hemoglobin, blood gas, and rheology were remarkably improved. The course of COPD is long and occurs repeatedly. Only when patients master the relevant professional knowledge of COPD, they can fundamentally establish healthy behavior and delay the progress of the disease [45–47].

In this study, nursing satisfaction based on knowledge, belief, and practice mode was remarkably higher when compared to routine department nursing, which fully confirmed the superiority of knowledge, belief, and practice mode of health education. Nursing quality and nursing effect were better, and it is more and more recognized by patients, and its application prospect is broader. The scores of nurse-led health education based on knowledge, belief, and practice model in all dimensions of KAP were remarkably higher than those in routine department nursing. Based on the model of knowledge, belief, and practice, nurse-led health education showed significant improvement in treatment compliance and self-management, which is closely related to improved KAP score. Awareness of the disease can affect the subjective initiative of patients, which contributes to improving their lung function. As an important index of disease change, life quality naturally improves after lung function is improved. As can be seen, the above indicators are related to each other. The same idea can be found in the study put forward by Meng and Yu [48]. They have applied new methods in the study, and the conclusions drawn can also give some support to this study.

To sum up, nurse-led health education model based on knowledge, belief, and practice can successfully enhance the self-management ability, satisfaction, and compliance of elderly COPD patients. Our results suggest that nurse-led health education model based on knowledge, belief, and practice may be a reliable model for the management of COPD patients after treatment.

## Figures and Tables

**Figure 1:** 

**Figure 2:** 

**Table 1:** KAP scores between the two groups ($\bar{x}\pm s$, points).

Group	*N*	Knowledge				Attitude				Behavior			
		Before nursing	After nursing	*t*	*P*	Before nursing	After nursing	*t*	*P*	Before nursing	After nursing	*t*	*P*
C group	30	10.84 ± 2.31	11.29 ± 1.55	0.886	>0.05	2.85 ± 1.21	3.39 ± 1.66	1.440	>0.05	2.58 ± 1.33	2.49 ± 0.21	0.366	>0.05
R group	30	10.89 ± 2.44	12.59 ± 2.12	2.881	<0.05	2.81 ± 1.34	4.84 ± 2.21	4.302	<0.01	2.59 ± 1.54	4.39 ± 1.21	5.034	<0.01
*t*		0.081	2.711			0.121	2.873			0.026	8.473		
*P*		>0.05	<0.01			>0.05	<0.01			>0.05	<0.01		

**Table 2:** The self-management level before and after nursing ($\bar{x}\pm s$, points).

Group	*N*	Symptom management		Daily life management		Emotion management		Information management		Management efficiency	
		Before nursing	After nursing	Before nursing	After nursing	Before nursing	After nursing	Before nursing	After nursing	Before nursing	After nursing
C group	30	22.77 ± 1.00	27.93 ± 0.42^∗^	23.50 ± 1.14	27.49 ± 1.21^∗^	24.40 ± 1.11	29.49 ± 1.21^∗^	17.77 ± 2.01	21.85 ± 3.31^∗^	16.91 ± 2.33	21.95 ± 2.64^∗^
R group	30	23.01 ± 1.05	29.93 ± 1.21^∗^	23.79 ± 1.24	31.29 ± 1.35^∗^	24.77 ± 1.23	34.19 ± 2.43^∗^	17.95 ± 2.21	26.94 ± 2.44^∗^	16.01 ± 2.40	25.49 ± 4.32^∗^
*t*		0.907	8.552	0.943	11.480	1.223	9.483	0.330	6.779	1.474	3.829
*P*		>0.05	<0.01	>0.05	<0.01	>0.05	<0.01	>0.05	<0.01	>0.05	<0.01

^∗^Compared with before nursing (*P* < 0.05).

**Table 3:** The pulmonary function between the two groups ($\bar{x}\pm s$).

Group	*N*	6 min walking distance (m)		FEV1%		FEV1/FVC%	
		Before nursing	After nursing	Before nursing	After nursing	Before nursing	After nursing
C group	30	284.54 ± 53.12	389.92 ± 18.42^∗^	45.91 ± 3.12	50.91 ± 3.36^∗^	48.93 ± 3.31	50.93 ± 3.36^∗^
R group	30	285.93 ± 53.55	405.92 ± 23.24^∗^	45.92 ± 3.44	59.49 ± 2.45^∗^	48.59 ± 3.56	55.91 ± 2.21^∗^
*t*		0.100	2.955	0.011	11.301	0.383	6.782
*P*		>0.05	<0.01	>0.05	<0.01	>0.05	<0.01

^∗^Compared with before nursing (*P* < 0.05).

**Table 4:** The life quality scores before and after nursing ($\bar{x}\pm s$, points).

Group	*N*	Physiological function		Psychological function		Social function		Healthy self-cognition	
		Before nursing	After nursing	Before nursing	After nursing	Before nursing	After nursing	Before nursing	After nursing
C group	30	15.42 ± 4.74	13.64 ± 2.55^∗^	16.66 ± 3.23	14.46 ± 1.55^∗^	18.82 ± 3.95	16.13 ± 2.45^∗^	15.34 ± 3.44	13.56 ± 1.85^∗^
R group	30	15.77 ± 4.42	11.84 ± 2.33^∗^	16.65 ± 3.21	12.81 ± 1.85^∗^	18.55 ± 3.46	12.84 ± 3.19^∗^	15.87 ± 3.72	10.83 ± 2.81^∗^
*t*		0.295	2.854	0.012	3.744	0.281	4.480	0.572	4.444
*P*		>0.05	<0.01	>0.05	<0.01	>0.05	<0.01	>0.05	<0.01

^∗^Compared with before nursing (*P* < 0.05).

## Data Availability

The datasets used and analyzed during the current study are available from the corresponding author upon reasonable request.
